The article "Systematic Characterization of Expression Patterns and Immunocorrelations of Formin-Like Genes in Breast Cancer" was published in 2022. Journal: Biomed Res Int.

# Systematic Characterization of Expression Patterns and Immunocorrelations of Formin-Like Genes in Breast Cancer

**DOI:** 10.1155/2022/8577821

**Published:** 2022-09-10

**Authors:** Erli Gao, Xuehai Wang, Fengxu Wang, Siyuan Deng, Weiyi Xia, Rui Wang, Xiangdong Wang, Xinyuan Zhao, Haixin Qian

**Affiliations:** ^1^Department of General Surgery, The First Affiliated Hospital of Soochow University, 188 Shizi Street, Shi Zi Road, Gusu District, Jiangsu, 215006, Suzhou, China; ^2^Department of Occupational Medicine and Environmental Toxicology, Nantong Key Laboratory of Environmental Toxicology, School of Public Health, Nantong University, Nantong 226019, China

## Abstract

**Background:**

Members of the formin-like gene (FMNL) family are required for cytoskeleton-related processes, and their expressions are implicated to the progression of a multitude of malignancies. However, there are insufficient studies on transcription factors and promising prognosis benefit of FMNLs during the genesis of breast cancer (BrCa).

**Methods:**

The transcriptional levels of FMNL family members in primary BrCa tissues and their association with intrinsic subclasses were analyzed using the UALCAN database. Then, the prognostic values of FMNLs in BrCa patients were investigated via the Kaplan-Meier plotter. Moreover, the correlations between FMNL expression levels and immune infiltrations were analyzed using the TIMER database. In addition, the expression patterns of FMNLs in BrCa were investigated by single-cell RNA-sequencing (scRNA-seq) analysis and were validated by immunohistochemistry (IHC) staining.

**Results:**

The transcriptional level of FMNL1 was shown to be considerably increased in BrCa. It is surprising that the transcriptional quantities of FMNL2 and FMNL3 were substantially reduced. In addition, during the comparison of several BrCa subclasses, FMNL1 and FMNL2 mRNA levels of patients with HER2-positive and triple-negative BrCa subclasses increased, while FMNL3 mRNA levels reduced. With the processions of experimentation, high FMNL1 expression was hopefully linked to well clinical outcome, while high FMNL2 expression predicted poor prognosis. Moreover, FMNL1 was highly expressed in tumor-infiltrating immune cells (TIICs) in tumor tissues. Last but not least, FMNL1 was highly expressed in TIICs and served as a gene marker for TIICs.

**Conclusions:**

The fact and result which we analyzed demonstrate FMNL1 as a diagnostic marker for TIICs by comprehensively elucidating the expression patterns and changeable prognostic implications of FMNLs in BrCa clinical applications.

## 1. Introduction

Breast cancer (BrCa) is the one of the most common cancers in middle-aged and older female [1]. It will be diagnosed in 12% of women in the United States over the course of their lifetimes, and more than 250,000 new cases of BrCa were diagnosed in the United States in 2017 [2]. It accounts for about 30% of all new cancers in women each year. According to American Cancer Society's estimates for BrCa in the United States for 2022, about 287,850 new cases of invasive BrCa will be diagnosed in women [3]. About 51,400 new cases of ductal carcinoma in situ (DCIS) will be diagnosed [4]. BrCa is the second major cause of cancer death in femme (lung cancer is the leading cause of cancer death in women). The chance that a woman will die from BrCa is about 2.6% [5].

The article "Systematic Characterization of Expression Patterns and Immunocorrelations of Formin-Like Genes in Breast Cancer" was published in 2022. Journal: Biomed Res Int.

Comprehensive therapies for breast cancer include biological targeting agents, systemic chemotherapeutic, less deviations radiotherapy, endocrine regulation and stimulation therapy, locoregional surgery, and a multidimension of the combination as those mentioned above, mainly depending on therapeutics, morphological, and chromosomal level consideration [6]. Biomarkers are mostly served as proxy of those therapies for constructing possibly life-threatening and forecasting the consequence in detail [7]. As just a conclusion, the improvement of more reliable and durable biomarkers for the prognosis of cancer patients has been recognized as the key to a breakthrough in cancer awareness [8]. Formin-like protein genes (FMNLs), the novel biomarkers in the prognostic predication, have performed promising correlations between high-level expression and better prognostic outcome [9]. Therefore, a sustainable analysis is anticipated that contained the data analysis and immunochemistry experiment to verify whether FMNLs could become a novel biomarker for BrCa.

In this research, we drove several scripts as a bioinformatic visualization and calculation of the clinical samples and tissue optical feature as it had been linked to FMNLs in BrCa access to online databases which contains large cohort and high credibility, evaluating the prognostic value of FMNL expression level in the treatment strategies of breast cancer [10]. Overall, our research preliminarily but systematically characterized the expression profiles of FMNLs in BrCa and revealed that the detection of the FMNL expression status of BrC patients may be valuable and potential biomarkers for prognostic assessment.

## 2. Methods

### 2.1. UALCAN Database Analysis

The UALCAN tool (http://ualcan.path.uab.edu/) is a level 3 RNA-seq online open-access platform [11] from the TCGA database. It can be used to compare the genes of perspective impetus between malignant and normal tissues at transcriptional levels, as well as the correlation between transcriptional levels and clinicopathologic characteristics. UALCAN was used to examine the transcriptome frequencies of FMNL family members in primary BrCa tissues and associated relationships between intrinsic subclasses in the current investigation. Our paper examined all the BrCa cases available on UALCAN.

The article "Systematic Characterization of Expression Patterns and Immunocorrelations of Formin-Like Genes in Breast Cancer" was published in 2022. Journal: Biomed Res Int.

### 2.2. Kaplan-Meier Plotter

The Kaplan-Meier Plotter (KM Plotter, http://kmplot.com/analysis/) database is an online database that contains gene expression profiles and survival data of cancer suffers [12]. All BrCa samples accessible on KM Plotter were used to investigate the prognostic values of FMNLs in BrCa. The patients were divided into cohorts based on the median expression of each FMNL's mRNA level. KM survival plots were used to compare all cohorts. The log-rank *P* value, hazard ratio (HR), and 95 percent confidence interval (95% CI) were computed and shown online.

### 2.3. Linked Omics Database Analysis

The Linked Omics database (http://www.linkedomics.org/login.php) is a web-based tool for examining and evaluating multidimensional datasets [13]. By gene set enrichment analysis, the functional functions of FMNLs in breast cancer were anticipated using the Linked Omics software in terms of Gene Ontology (GO) and Kyoto Encyclopedia of Genes and Genomes (KEGG) analyses (GSEA). For all parameters, the default choices were utilized.

### 2.4. TIMER Database Analysis

The TIMER database (http://cistrome.shinyapps.io/timer/) may be used to analyze gene expression and immune infiltration across various cancer types [14]. The following were the screening conditions for immunological infiltration of the submitted FMNLs in BrCa: (1) cancer type: breast cancer and (2) immune infiltrates: B cell, CD8+ T cell, CD4+ T cell, macrophage, neutrophil, and dendritic cell.

### 2.5. TISCH Database Analysis

TME is the focus of the TISCH database (http://tisch.comp-genomics.org), which is a scRNA-seq database [15]. The TISCH tool provides detailed cell type annotation at the single-cell level, facilitating TME investigation across many cancer types. The TISCH software generates a dot plot that illustrates the intensity of marker gene expression including all identified types of cells.

### 2.6. HPA Database Analysis

The Human Protein Atlas (HPA) is a program which combines microscopy, proteomics, and transcriptomics to classify human proteins. The HPA information can be acquired primarily through a web-based interface that allows individual protein inspections, which may not be appropriate for gene set data analysis or automatic retrieval of original images.

### 2.7. Clinical Samples

The BrCa tissue microarray (TMA, Cat. HBre-Duc060CS-03) was obtained from Outdo Biotech (Shanghai, China). The TMA contained 30 tumor samples and 30 paired adjacent samples. Detailed clinicopathological characteristics of the cohorts were provided by Outdo Biotech. The tissue microarray was submitted for immunohistochemistry (IHC) staining in this research. Ethical approval (YB-M-05-02) for the study of TMA was granted by the Clinical Research Ethics Committee, Outdo Biotech (Shanghai, China).

The article "Systematic Characterization of Expression Patterns and Immunocorrelations of Formin-Like Genes in Breast Cancer" was published in 2022. Journal: Biomed Res Int.

### 2.8. Immunohistochemistry Staining

Standard techniques were used to do IHC staining on the HBre-Duc060CS-03 TMA. Anti-FMNL1 (1 : 800 dilution, Cat. 27834-1-AP, Proteintech, Wuhan, China) and anti-PD-L1 were utilized as primary antibodies (ready-to-use, Cat. GT2280, GeneTech, Shanghai, China). DAB and hematoxylin counterstain were used to visualize antibody staining, and stained sections were imaged using Aperio Digital Pathology Slide Scanners. The stained sections were examined separately by two pathologists according to the assessment criteria on a 12-point scale by generating the immunoreactivity score (IRS) for semiquantitative analysis [16]. The percentage of positively stained cells was scored as 0–4: 0 (<5%), 1 (6–25%), 2 (26–50%), 3 (51–75%), and 4 (>75%). The staining intensity was scored as 0–3: 0 (negative), 1 (weak), 2 (moderate), and 3 (strong). The immunoreactivity score (IRS) equals to the percentages of positive cells multiplied with staining intensity.

### 2.9. Statistical Analysis

All statistical analyses were carried out through the internet utilizing appropriate bioinformatics websites. The Student *t*-test was used to analyze for abnormalities in FMNL expression, Pearson's test was utilized for gene expression and immune cell infiltration association analysis, and the log-rank test was employed for survival analysis. Distinctions were deemed statistically significant in all analyses if the *P* value was < 0.05.

## 3. Results

### 3.1. Differential Expression of FMNLs in BRCA and Normal Breast Tissues

To assess the exact expression profiles of FMNL family members in BrCa patients, the UALCAN database was used to assess differences in transcriptional levels of FMNL family members between BrCa and paired normal breast tissue. The transcriptional level of FMNL1 was significantly upregulated in BrCa tissues compared with paracancerous tissues (Figure 1(a)). However, the transcriptional levels of FMNL2 and FMNL3 were dramatically downregulated in BrCa tissues compared with paracancerous tissues (Figures 1(b) and 1(c)). The protein levels of FMNL1 (Figure 1(d)) and FMNL3 (Figure 1(f)) were significantly upregulated in BrCa tissues compared with paracancerous tissues, but the protein level of FMNL2 (Figure 1(e)) was significantly downregulated in BrCa tissues compared with paracancerous tissues. Above all, we made different expressions of FMNLs in the different stages, and we can see the differences between different stages of tumors. Comparing the expression of FMNL1 in the normal tissues and cancer tissues, the stages 1, 2, and 3 have great difference to the normal tissues (Figure 2(a)). Comparing the expression of FMNL2 in the normal tissues and cancer tissues, not only the stages 1, 2, 3, and 4 have the great difference to the normal tissues, but also the FMNL2 has the difference between stage 2 and stage 3 (Figure 2(b)). There is no significant difference in the expression of FMNL3 in the normal tissues and cancer tissue, while we can find only that stage 1 and stage 2 have the difference, which could not give the direct evidence to prove the FMNL3 has effect on the different stages of the breast cancer (Figure 2(c)). But the analysis gives us a probability that the FMNL1 and FMNL2 mediate tumorigenesis and progress.

The article "Systematic Characterization of Expression Patterns and Immunocorrelations of Formin-Like Genes in Breast Cancer" was published in 2022. Journal: Biomed Res Int.

### 3.2. Associations of FMNL Expressions with the Molecular Subtypes of BRCA

Classification of intrinsic subclasses is helpful in the prediction of therapeutic response and prognosis of BrCa [17]. So, we next compared the differential transcriptional levels of FMNL family members according to different intrinsic subclasses of BrCa. The mRNA expressions of FMNL family members were significantly correlated with intrinsic subclasses of BrCa. Patients who were with HER2-positive and triple-negative BrCa tended to express higher FMNL1 and FMNL2 mRNA levels (Figures 3(a), 3(b), 3(d), and 3(e)) while expressed lower FMNL3 mRNA (Figures 3(c) and 3(f)). By combining the mRNA expression and protein expression for each gene, we can find that the FMNL1 mRNA has highest expression in the TNBC, the worst subtype of BRCA (Figure 2(a)). Moreover, we find that the FMNL1 protein expression in TNBC is lower than the HER2 positive interestingly (Figure 2(d)). This fact may suggest there is something interrupting the mRNA translation during the TNBC genesis and progress. For FMNL2, 3 mRNA, and protein expressions, the same momentum happens, mRNA expressions different but proteins' average (Figures 2(e) and 2(f)). The situation needs more research on it.

### 3.3. Prognostic Values of FMNLs in BRCA

Furthermore, we employed the KM Plotter to evaluate the prognostic values of FMNL family members. As the HR goes up, we can see that the survival rate goes up, and higher mRNA expression of FMNL1 also resulted in increased survival rate (Figures 4(a), 4(d), and 4(g)), and FMNL2 (Figures 4(b), 4(e), and 4(h)) was significantly associated with better probability of BrCa patients. By contrast, the mRNA expression of FMNL3 was not significantly correlated with the prognosis with the increase of HR but showed a certain correlation on the whole (Figures 4(c), 4(f), and 4(i)). In summary, we found that FMNL1 was highly expressed in tumors but was associated with better prognosis.

The article "Systematic Characterization of Expression Patterns and Immunocorrelations of Formin-Like Genes in Breast Cancer" was published in 2022. Journal: Biomed Res Int.

### 3.4. Biological Roles of FMNLs in BRCA

Subsequently, we carried out GO analysis, including biological process (BP), cellular component (CC), molecular function (MF) analysis, and KEGG analysis, on FMNLs and their interacting genes using the DAVID platform. Moreover, results from the Linked Omics database revealed that FMNLs participate in many immune processes. Tables 1–3 exhibited the top 5 most highly enriched GO and KEGG terms. High expression of FMNL1 was associated with respiratory burst, leukocyte apoptotic process, positive regulation of cell activation, interleukin-4 production, mast cell activation (BP category), MHC protein complex, immunological synapse, endoplasmic reticulum tubular network, mast cell granule, protein complex involved in cell adhesion (CC category), MHC protein binding, antigen binding, nucleotide receptor activity, cytokine receptor activity, pattern recognition receptor activity (MF category), graft-versus-host disease, autoimmune thyroid disease, allograft rejection, type I diabetes mellitus, and Staphylococcus aureus infection (KEGG category). High expression of FMNL2 was associated with adaptive immune response, leukocyte proliferation, positive regulation of cell activation, leukocyte cell-cell adhesion, immune response-regulating signaling pathway (BP category), mitochondrial membrane part, NADH dehydrogenase complex, mitochondrial inner membrane, mitochondrial protein complex, respiratory chain (CC category), cytokine binding, cytokine receptor activity structural constituent of ribosome, hijacked molecular function, coreceptor activity (MF category), cytokine-cytokine receptor interaction, leishmaniasis, osteoclast differentiation, hematopoietic cell lineage, and measles (KEGG category). High expression of FMNL3 was associated with RNA capping, DNA damage response, detection of DNA damage, NADH dehydrogenase complex assembly, mitochondrial respiratory chain complex assembly, metallo-sulfur cluster assembly (BP category), nucleoid, chaperone complex, small nucleolar ribonucleoprotein complex, cytochrome complex, NADH dehydrogenase complex (CC category), nucleotide receptor activity, purinergic receptor activity, coreceptor activity, extracellular matrix structural constituent, threonine-type peptidase activity (MF category), aminoacyl-tRNA biosynthesis, protein export, terpenoid backbone biosynthesis, nucleotide excision repair, and RNA polymerase (KEGG category). Taken together, GO and KEGG analyses revealed the potential molecular mechanisms of FMNLs in BrCa.

The article "Systematic Characterization of Expression Patterns and Immunocorrelations of Formin-Like Genes in Breast Cancer" was published in 2022. Journal: Biomed Res Int.

### 3.5. Relationship between the Expression of FMNLs and Immune Infiltration in BRCA

Tumor-infiltrating immune cells (TIICs) are independent predictors of the sentinel lymph node status and cancer survival [18, 19]. Therefore, our study further evaluated the correlation between FMNL expressions and immune infiltration in BrCa using the TIMER database. The results showed that the expression of FMNL1 was positively correlated with the infiltration levels of B cells, CD8+ T cells, CD4+ T cells, macrophages, neutrophils, and dendritic cells in BrCa (Figure 5(a)). FMNL2 was positively correlated with the infiltration levels of B cells, CD8+ T cells, CD4+ T cells, macrophages, neutrophils, and dendritic cells in BrCa (Figure 5(a)). Additionally, FMNL3 had a positive correlation with the infiltrating levels of B cells, CD8+ T cells, CD4+ T cells, macrophages, neutrophils, and dendritic cells in BrCa (Figure 5(a)). But all three were negatively correlated with tumor purity (Figures 5(a)–5(c)). These results strongly suggested that FMNLs played specific roles in regulating immune infiltration in BrCa.

### 3.6. The Analysis of the Correlation between the FMNLs and the Immune Cell Markers

Considering the specificity of FMNLs in the immune microenvironment, the family member may be immune cell markers to a certain extent. So we carried out correlation analysis of immune cell subtypes to further exploration. As shown in Table 4, we evaluated the correlation between FMNL1 and immune cell subtypes in breast cancer and found that it was positively correlated with the vast majority of immune cell subtypes but negatively with the gene marker GATA3 in TH2 cells, demonstrating the worse prognosis of BrCa and high correlation of the immunotherapy of PD-L1 and CTLA4.

### 3.7. Analysis of FMNL Expression Cell Subpopulations in BRCA

The TISCH tool provides a dot plot to show marker gene expression levels for all annotated cell types. The expression abundance of FMNL1 was significantly higher than that of FMNL2 and FMNL3, and FMNL1 was highly expressed in immune cells (Figures 6(a)–6(d)). Therefore, we speculated that FMNL1 expression from bulk RNA-seq was derived from TIICs, which might explain that high FMNL1 expression was associated with a better prognosis in BrCa.

Additionally, we also validated the expression patterns of FMNLs using IHC staining. In the HPA database, we found that FMNL1 was highly detected in TIICs (Figure 7(a)), while FMNL2 and FMNL3 were lowly expressed in all cell types in BrCa (Figures 7(b) and 7(c)). Moreover, the in-house cohort was also used to validate our current finding. The results showed that FMNL1 was highly expressed in TIICs as well (Figure 7(d)). The difference of PD-L1 between high and low FMNL groups was detected because FMNL1 is a marker of tumor-infiltrating immune cells, and tumors with many immune cells are hot tumors. Therefore, FMNL1 can be considered as a marker of hot tumors, while PD-L1 is upregulated in hot tumors. Moreover, the current BrCa cohort was segregated into low and high FMNL1 expression groups, and we observed that PD-L1 was overexpressed in the high FMNL1 group (Figure 7(e)). Overall, these results revealed that FMNL1 is highly expressed in TIICs in BrCa, which might account for the contradictory correlation between expression status and prognosis value.

The article "Systematic Characterization of Expression Patterns and Immunocorrelations of Formin-Like Genes in Breast Cancer" was published in 2022. Journal: Biomed Res Int.

### 3.8. The Correlation between FMNLs and Immune Checkpoints

In order to further understand its role in TME, we performed immune checkpoint correlation analysis on FMNL family members (Table 5). In our analysis of 23 immune checkpoints, we can clearly find that FMNL1 was positively correlated with it, and the correlation of target PD-1 was especially positive in the ICB treatment, which is widely used today. Furthermore, the strong positive correlation of CTLA-4 will provide predictions for assessing immune cell performance in the context of emerging therapy CAR-T. But FMNL2 was only negatively correlated with ADORA2A, and FMNL3 was only negatively correlated with PVR. This further confirmed our conjecture because at first, in the systematic analysis of the expression and prognosis of FMNL1-3 in breast cancer, we found that FMNL1 was highly expressed in tumors but was associated with better prognosis, so it was not in line with the routine, which proved that FMNL1 acted as an immune cell marker.

## 4. Discussion

Bioinformatics has recently seen a surge in immune interaction analysis of candidates [20]. However, fewer specific analyses had been performed, and a vast percentage of substandard analyses had been unable to draw substantiate results. In the previous study, we found that FMNL1 influences prognosis tremendously in non-small-cell lung cancer (NSCLC) by its expression [21], but without valid research continuing. FMNL1 was discovered to be a novel biomarker for immune cells in our study, based on public data and biological confirmation. In regular analysis of bulk RNA-seq data, obvious immunocorrelations could be seen due to its certain expression pattern. FMNL1 is a member of the formin protein family that assists in membrane polymerization [22]. FMNL1 is a component of the diaphanous-related formins (DRF) subfamily of formins, which is involved in phagocytosis, cell adhesion, podosome dynamics, cell migration, cytokinesis, and polarity control. FMNL1 expression was shown to be upregulated in a variety of cancers, and this upregulation aided cell invasiveness. FMNL1 could intensify the aggressiveness of tumor cells intensify the aggressiveness of tumor cells through a variety of ways, in addition to facilitating cytoskeletal remodeling [23]. FMNL1 increased cell aggressiveness in nasopharyngeal cancer by epigenetically upregulating MTA1. FMNL1 inhibition inhibits bone metastases in NSCLC via inhibiting TGF-1 signaling [21].

The article "Systematic Characterization of Expression Patterns and Immunocorrelations of Formin-Like Genes in Breast Cancer" was published in 2022. Journal: Biomed Res Int.

FMNL1 is primarily expressed in immune cells and tissues such as clear cell renal cell carcinoma and the nasopharyngeal carcinoma [24, 25], despite its role as a critical oncogene in a variety of cancers. FMNL1 is highly expressed in lymphoid and myeloid leukemias, nonlymphomas, Hodgkin's, and malignant lymphoid and myeloid cell lines [26, 27], among other hematopoietic malignancies. The tumor mass, as we all know, is complex, containing both cancerous and antitumor immune cells. Because FMNL1 is highly expressed in immune cells rather than tumor cells, the expression of FMNL1 mRNA in tumor tissues is derived primarily from TIICs using bulk RNA-seq analysis. As a result, the expression of bulk FMNL1 mRNA was highly immunoreacted.

In the current study, we discovered that high FMNL1 expression predicted a better prognosis in HCC. Previous studies have linked high FMNL1 expression to a poor prognosis in a variety of cancers, including clear cell renal cell carcinoma [23], gastric cancer [9], and glioblastoma [28]. FMNL1 was found to promote T cell and macrophage migration in the previous studies [29, 30]. As a result, we hypothesized that FMNL1+ immune cells had a higher level of ability to migrate, making them more likely to play anti-tumor roles. FMNL1 was also found in tumor cells, indicating that it functions as a critical oncogene in a variety of cancers [9]. As a result, we hypothesized that the balance of FMNL1 expression in tumor and immune cells resulted in different prognostic phenotypes in various cancers.

## 5. Conclusions

Consequently, the immunological association and cell subpopulation transcriptome pattern of FMNL1 were studied in detailed. Despite the fact that FMNL1 was inherently related to immune infiltration, it was only a new marker for immune cells. To avoid being misled by bulk RNA-seq datasets, blind immune infiltration analyses should be further confirmed using scRNA-seq or IHC.

## Figures and Tables

**Figure 1:** Expression levels of FMNLs in paracancerous and BrCa tissues. (a) The transcriptional level of FMNL1 was upregulated in BrCa tissues compared with paracancerous tissues. (b, c) The transcriptional levels of FMNL2 and FMNL3 were downregulated in BrCa tissues compared with paracancerous tissues. (d, f) The protein levels of FMNL1 and FMNL3 were upregulated in BrCa tissues compared with paracancerous tissues. (e) The protein level of FMNL2 was downregulated in BrCa tissues compared with paracancerous tissues.

The article "Systematic Characterization of Expression Patterns and Immunocorrelations of Formin-Like Genes in Breast Cancer" was published in 2022. Journal: Biomed Res Int.

**Figure 2:** Associations between FMNL expression levels and molecular subtypes of BrCa. (a–c) The FMNL member mRNA expression on individual cancer stages from TCGA samples. (d–f) The FMNL member protein expressions on individual cancer stages from CPTAC samples.

**Figure 3:** Associations between FMNL expression levels and molecular subtypes of BrCa. (a–c) The transcriptional level of FMNLs in normal breast tissues and BrCa tissues with different intrinsic subclasses. (d, e) The protein level of FMNLs in normal breast tissues and BrCa tissues with different intrinsic subclasses.

**Figure 4:** The prognostic values of FMNLs in patients with BrCa. (a, d, g) High mRNA levels of FMNL1 were related with poor OS, RFS, and DMFS in BrCa. (b, e, h, c, f, i) The FMNL2&3 mRNA level had no obvious relation with OS, RFS, and DMFS in BrCa. OS: overall survival; RFS: relapse-free survival; DMFS: distant metastasis-free survival. Color images are available online.

**Figure 5:** Correlations of FMNL expression with immune infiltrating level in BrCa. (a–c) FMNL1-3 expressions were significantly negatively related to tumor purity while positively correlated with infiltrating levels of CD8+ T cells, CD4+ T cells, macrophages, neutrophils, and DCs in GC. DC: dendritic cell. Color images are available online.

**Figure 6:** The dot plots showed the expression patterns of FMNLs generated by TISCH. (a) The scRNA-seq data from the GSE136206 dataset. (b) The scRNA-seq data from the GSE114727 dataset. (c) The scRNA-seq data from the GSE143423 dataset. (d) The scRNA-seq data from the GSE114727 dataset.

**Figure 7:** Protein expression of FMNLs detected by IHC in BrCa. (a–c) FMNL protein levels in BRCA were visualized by IHC in HPA. (d) Representative microphotographs revealing low and high FMNL1 and PD-L1 expressions using IHC staining. (e) PD-L1 expression in the low and high FMNL1 groups in BrCa.

**Table 1:** GO and KEGG pathway enrichment analyses of FMNL1 in BRCA.

Term	Description	Size	NES	FDR
Biological process				
GO:0045730	Respiratory burst	27	1.524	0.005
GO:0071887	Leukocyte apoptotic process	103	1.488	0.005
GO:0050867	Positive regulation of cell activation	298	1.490	0.005
GO:0032633	Interleukin-4 production	34	1.504	0.005
GO:0045576	Mast cell activation	58	1.502	0.005
Cell component				
GO:0042611	MHC protein complex	19	1.581	<0.001
GO:0001772	Immunological synapse	32	1.558	<0.001
GO:0071782	Endoplasmic reticulum tubular network	18	-2.144	<0.001
GO:0042629	Mast cell granule	21	1.503	0.001
GO:0098636	Protein complex involved in cell adhesion	35	1.517	0.001
Molecular function				
GO:0042287	MHC protein binding	24	1.563	<0.001
GO:0003823	Antigen binding	52	1.536	<0.001
GO:0016502	Nucleotide receptor activity	22	1.495	0.011
GO:0004896	Cytokine receptor activity	88	1.476	0.012
GO:0038187	Pattern recognition receptor activity	20	1.477	0.015
KEGG				
hsa05332	Graft-versus-host disease	37	1.616	<0.001
hsa05320	Autoimmune thyroid disease	50	1.608	<0.001
hsa05330	Allograft rejection	35	1.591	<0.001
hsa04940	Type I diabetes mellitus	41	1.588	<0.001
hsa05150	Staphylococcus aureus infection	52	1.584	<0.001

Note: NES: normalized enrichment score.

The article "Systematic Characterization of Expression Patterns and Immunocorrelations of Formin-Like Genes in Breast Cancer" was published in 2022. Journal: Biomed Res Int.

**Table 2:** GO and KEGG pathway enrichment analyses of FMNL2 in BRCA.

Term	Description	Size	NES	FDR
Biological process				
GO:0002250	Adaptive immune response	368	2.101	<0.001
GO:0070661	Leukocyte proliferation	274	2.047	<0.001
GO:0050867	Positive regulation of cell activation	298	2.007	<0.001
GO:0007159	Leukocyte cell-cell adhesion	310	2.004	<0.001
GO:0002764	Immune response-regulating signaling pathway	452	2.004	<0.001
Cell component				
GO:0044455	Mitochondrial membrane part	167	-2.188	<0.001
GO:0030964	NADH dehydrogenase complex	43	-2.292	<0.001
GO:0005743	Mitochondrial inner membrane	369	-2.305	<0.001
GO:0098798	Mitochondrial protein complex	213	-2.338	<0.001
GO:0070469	Respiratory chain	84	-2.387	<0.001
Molecular function				
GO:0019955	Cytokine binding	119	1.987	<0.001
GO:0004896	Cytokine receptor activity	88	1.938	<0.001
GO:0003735	Structural constituent of ribosome	153	-2.251	<0.001
GO:0104005	Hijacked molecular function	70	1.834	0.001
GO:0015026	Coreceptor activity	39	1.810	0.002
KEGG				
hsa04060	Cytokine-cytokine receptor interaction	281	2.016	<0.001
hsa05140	Leishmaniasis	71	1.961	<0.001
hsa04380	Osteoclast differentiation	126	1.944	<0.001
hsa04640	Hematopoietic cell lineage	93	1.916	<0.001
hsa05162	Measles	129	1.911	<0.001

Note: NES: normalized enrichment score.

**Table 3:** GO and KEGG pathway enrichment analyses of FMNL3 in BRCA.

Term	Description	Size	NES	FDR
Biological process				
GO:0036260	RNA capping	30	-2.131	<0.001
GO:0042769	DNA damage response, detection of DNA damage	38	-2.134	<0.001
GO:0010257	NADH dehydrogenase complex assembly	49	-2.838	<0.001
GO:0033108	Mitochondrial respiratory chain complex assembly	68	-3.256	<0.001
GO:0031163	Metallo-sulfur cluster assembly	17	-2.008	0.005
Cell component				
GO:0009295	Nucleoid	36	-2.024	<0.001
GO:0101031	Chaperone complex	21	-2.123	<0.001
GO:0005732	Small nucleolar ribonucleoprotein complex	20	-2.366	<0.001
GO:0070069	Cytochrome complex	29	-2.483	<0.001
GO:0030964	NADH dehydrogenase complex	43	-2.712	<0.001
Molecular function				
GO:0016502	Nucleotide receptor activity	22	1.646	<0.001
GO:0035586	Purinergic receptor activity	26	1.597	<0.001
GO:0015026	Coreceptor activity	39	1.589	<0.001
GO:0005201	Extracellular matrix structural constituent	151	1.570	<0.001
GO:0070003	Threonine-type peptidase activity	21	-2.285	<0.001
KEGG				
hsa00970	Aminoacyl-tRNA biosynthesis	43	-2.107	<0.001
hsa03060	Protein export	22	-2.120	<0.001
hsa00900	Terpenoid backbone biosynthesis	22	-2.132	<0.001
hsa03420	Nucleotide excision repair	45	-2.164	<0.001
hsa03020	RNA polymerase	31	-2.193	<0.001

Note: NES: normalized enrichment score.

The article "Systematic Characterization of Expression Patterns and Immunocorrelations of Formin-Like Genes in Breast Cancer" was published in 2022. Journal: Biomed Res Int.

**Table 4:** The correlation between FMNL and immune cell biomarkers.

Description	Gene marker	FMNL1		FMNL2		FMNL3	
		Correlation	*P* value	Correlation	*P* value	Correlation	*P* value
CD8+ T cell	CD8A	0.714	<0.001	0.397	<0.001	0.468	<0.001
	CD8B	0.663	<0.001	0.378	<0.001	0.355	<0.001
T cell (general)	CD3D	0.760	<0.001	0.373	<0.001	0.408	<0.001
	CD3E	0.759	<0.001	0.402	<0.001	0.460	<0.001
	CD2	0.762	<0.001	0.437	<0.001	0.466	<0.001
B cell	CD19	0.609	<0.001	0.280	<0.001	0.293	<0.001
	CD79A	0.595	<0.001	0.315	<0.001	0.327	<0.001
Monocyte	CD86	0.765	<0.001	0.566	<0.001	0.536	<0.001
	CSF1R	0.773	<0.001	0.479	<0.001	0.664	<0.001
TAM	CCL2	0.569	<0.001	0.446	<0.001	0.353	<0.001
	CD68	0.695	<0.001	0.493	<0.001	0.521	<0.001
	IL10	0.634	<0.001	0.491	<0.001	0.478	<0.001
M1 macrophage	NOS2	0.111	<0.001	0.286	<0.001	0.397	<0.001
	IRF5	0.589	<0.001	0.274	<0.001	0.333	<0.001
	PTGS2	0.293	<0.001	0.466	<0.001	0.395	<0.001
M2 macrophage	CD163	0.637	<0.001	0.545	0.000	0.462	<0.001
	VSIG4	0.545	<0.001	0.424	<0.001	0.429	<0.001
	MS4A4A	0.645	<0.001	0.528	<0.001	0.524	<0.001
Neutrophils	CEACAM8	0.015	0.624	0.090	0.003	0.015	0.630
	ITGAM	0.667	<0.001	0.399	<0.001	0.523	<0.001
	CCR7	0.692	<0.001	0.314	<0.001	0.414	<0.001
Natural killer cell	KIR2DL1	0.385	<0.001	0.278	<0.001	0.187	<0.001
	KIR2DL3	0.395	<0.001	0.265	<0.001	0.200	<0.001
	KIR2DL4	0.487	<0.001	0.346	<0.001	0.121	<0.001
	KIR3DL1	0.468	<0.001	0.320	<0.001	0.274	<0.001
	KIR3DL2	0.508	<0.001	0.309	<0.001	0.228	<0.001
	KIR3DL3	0.272	<0.001	0.176	<0.001	0.096	0.001
	KIR2DS4	0.356	<0.001	0.255	0.000	0.168	<0.001
Dendritic cell	HLA-DPB1	0.818	<0.001	0.314	<0.001	0.528	<0.001
	HLA-DQB1	0.666	<0.001	0.298	<0.001	0.363	<0.001
	HLA-DRA	0.784	<0.001	0.477	<0.001	0.571	<0.001
	HLA-DPA1	0.770	<0.001	0.429	<0.001	0.584	<0.001
	CD1C	0.583	<0.001	0.232	<0.001	0.498	<0.001
	NRP1	0.290	<0.001	0.448	<0.001	0.723	<0.001
	ITGAX	0.797	<0.001	0.509	<0.001	0.598	<0.001
Th1 cell	TBX21	0.759	<0.001	0.420	<0.001	0.432	<0.001
	STAT4	0.715	<0.001	0.479	<0.001	0.547	<0.001
	STAT1	0.450	<0.001	0.458	<0.001	0.304	<0.001
	IFNG	0.613	<0.001	0.432	<0.001	0.291	<0.001
	TNF	0.456	<0.001	0.334	<0.001	0.210	<0.001
Th2 cell	GATA3	*0.242*	<0.001	*0.483*	<0.001	*0.024*	0.426
	STAT6	0.216	<0.001	0.024	0.425	0.352	<0.001
	STAT5A	0.475	<0.001	0.257	<0.001	0.413	<0.001
	IL13	0.309	<0.001	0.257	<0.001	0.150	<0.001
Tfh cell	BCL6	0.145	<0.001	0.183	<0.001	0.301	<0.001
	IL21	0.429	<0.001	0.340	<0.001	0.250	<0.001
Th17 cell	STAT3	0.193	<0.001	0.292	<0.001	0.384	<0.001
	IL17A	0.239	<0.001	0.229	<0.001	0.102	0.001
Treg cell	FOXP3	0.682	<0.001	0.469	<0.001	0.422	<0.001
	CCR8	0.567	<0.001	0.513	<0.001	0.469	<0.001
	STAT5B	0.204	<0.001	0.164	<0.001	0.444	<0.001
	TGFB1	0.559	<0.001	0.189	<0.001	0.622	<0.001
Exhausted T cell	PDCD1	0.758	<0.001	0.354	0.000	0.319	<0.001
	CTLA4	0.702	<0.001	0.496	<0.001	0.343	<0.001
	LAG3	0.613	<0.001	0.349	<0.001	0.130	<0.001
	HAVCR2	0.705	<0.001	0.521	<0.001	0.569	<0.001
	GZMB	0.641	<0.001	0.439	<0.001	0.229	<0.001

PS: the italic characters are negatively correlated.

The article "Systematic Characterization of Expression Patterns and Immunocorrelations of Formin-Like Genes in Breast Cancer" was published in 2022. Journal: Biomed Res Int.

**Table 5:** The correlation between FMNL and immune checkpoints.

Immune checkpoint	FMNL1		FMNL2		FMNL3	
	Correlation	*P* value	Correlation	*P* value	Correlation	*P* value
VTCN1	0.100	0.001	0.171	<0.001	0.128	<0.001
CD274	0.561	<0.001	0.557	<0.001	0.506	<0.001
PDCD1	0.758	<0.001	0.354	<0.001	0.319	<0.001
CTLA4	0.702	<0.001	0.496	<0.001	0.343	<0.001
HAVCR2	0.705	<0.001	0.521	<0.001	0.569	<0.001
TIGIT	0.738	<0.001	0.501	<0.001	0.442	<0.001
IDO1	0.596	<0.001	0.487	<0.001	0.242	<0.001
CD80	0.582	<0.001	0.569	<0.001	0.424	<0.001
CD86	0.765	<0.001	0.566	<0.001	0.536	<0.001
LAIR1	0.805	<0.001	0.551	<0.001	0.607	<0.001
PVR	0.082	0.007	0.386	<0.001	*0.002*	0.957
CD200R1	0.690	<0.001	0.513	<0.001	0.652	<0.001
CD200	0.404	<0.001	0.460	<0.001	0.717	<0.001
LGALS3	0.202	<0.001	0.163	<0.001	0.226	<0.001
CEACAM1	0.086	0.004	0.212	<0.001	0.097	0.001
BTLA	0.687	<0.001	0.460	<0.001	0.476	<0.001
ADORA2A	0.341	<0.001	*0.010*	0.735	0.249	<0.001
KIR3DL1	0.468	<0.001	0.320	<0.001	0.274	<0.001
KLRC1	0.574	<0.001	0.380	<0.001	0.324	<0.001
CD276	0.145	<0.001	0.220	<0.001	0.311	<0.001
CD47	0.169	<0.001	0.404	<0.001	0.241	<0.001
KLRD1	0.632	<0.001	0.561	<0.001	0.500	<0.001
LAG3	0.613	<0.001	0.349	<0.001	0.130	<0.001

PS: the italic characters are negatively correlated.

## Data Availability

No data were used to support this study.

## References

[1] Belhadj A., Seddiki S., Belhadj A., Zakmout B., Araba A. E. K. A., Sahraoui T. (2021). Prevalence and prognosis of molecular phenotypes in breast cancer patients by age: a population-based retrospective cohort study in western Algeria. *The Pan African Medical Journal*.

The article "Systematic Characterization of Expression Patterns and Immunocorrelations of Formin-Like Genes in Breast Cancer" was published in 2022. Journal: Biomed Res Int.

[2] Ruiz-Casado A., Álvarez-Bustos A., de Pedro C. G., Méndez-Otero M., Romero-Elías M. (2021). Cancer-related fatigue in breast cancer survivors: a review. *Clinical Breast Cancer*.

[3] Siegel R. L., Miller K. D., Fuchs H. E., Jemal A. (2022). Cancer statistics, 2022. *CA: a Cancer Journal for Clinicians*.

[4] Weiss T., Loddenkemper R., Bittner R., Husen-Weiss E., Kaiser D., Felix R. (1988). Magnetic resonance tomography of the retro-stenotic syndrome. *Praxis und Klinik der Pneumologie*.

[5] Nixon N. A., Simmons C., Lemieux J., Verma S. (2020). Research priorities in metastatic breast cancer: a James Lind Alliance priority setting partnership. *The Breast Journal*.

[6] Yin L., Duan J. J., Bian X. W., Yu S. C. (2020). Triple-negative breast cancer molecular subtyping and treatment progress. *Breast Cancer Research*.

[7] Devos D., Moreau C., Kyheng M. (2019). A ferroptosis-based panel of prognostic biomarkers for amyotrophic lateral sclerosis. *Scientific Reports*.

[8] Doroshow D. B., Bhalla S., Beasley M. B. (2019). PD-L1 as a biomarker of response to immune-checkpoint inhibitors. *Nature reviews Clinical oncology*.

[9] Nie H., Mei J., Zhang Q., An F., Zhan Q. (2020). Systematic characterization of the expression and prognostic values of formin-like gene family in gastric cancer. *DNA and Cell Biology*.

[10] Manninen A. A., Gardberg M., Juteau S., Ilmonen S., Jukonen J., Andersson N. (2019). BRAF immunohistochemistry predicts sentinel lymph node involvement in intermediate thickness melanomas. *PloS one*.

[11] Chandrashekar D. S., Bashel B., Balasubramanya S. A. H. (2017). UALCAN: a portal for facilitating tumor subgroup gene expression and survival analyses. *Neoplasia (New York, NY)*.

[12] Lánczky A., Győrffy B. (2021). Web-based survival analysis tool tailored for medical research (KMplot): development and implementation. *Journal of Medical Internet Research*.

[13] Vasaikar S. V., Straub P., Wang J., Zhang B. (2018). LinkedOmics: analyzing multi-omics data within and across 32 cancer types. *Nucleic Acids Research*.

[14] Li T., Fan J., Wang B. (2017). TIMER: a web server for comprehensive analysis of tumor-infiltrating immune cells. *Cancer Research*.

[15] Sun D., Wang J., Han Y. (2021). TISCH: a comprehensive web resource enabling interactive single-cell transcriptome visualization of tumor microenvironment. *Nucleic Acids Research*.

[16] Mei J., Liu Y., Yu X. (2021). YWHAZ interacts with DAAM1 to promote cell migration in breast cancer. *Cell Death Discovery*.

[17] Sporikova Z., Koudelakova V., Trojanec R., Hajduch M. (2018). Genetic markers in triple-negative breast cancer. *Clinical Breast Cancer*.

The article "Systematic Characterization of Expression Patterns and Immunocorrelations of Formin-Like Genes in Breast Cancer" was published in 2022. Journal: Biomed Res Int.

[18] Grotz T. E., Vaince F., Hieken T. J. (2013). Tumor-infiltrating lymphocyte response in cutaneous melanoma in the elderly predicts clinical outcomes. *Melanoma Research*.

[19] Mei J., Yang X., Xia D. (2020). Systematic summarization of the expression profiles and prognostic roles of the dishevelled gene family in hepatocellular carcinoma. *Molecular Genetics & Genomic Medicine*.

[20] Tan Y. Q., Li Y. T., Yan T. F. (2020). Six Immune Associated Genes Construct Prognostic Model Evaluate Low-Grade Glioma. *Frontiers in immunology*.

[21] Yang X. Y., Liao J. J., Xue W. R. (2019). FMNL1 down-regulation suppresses bone metastasis through reducing TGF-*β*1 expression in non-small cell lung cancer (NSCLC). *Biomedicine & Pharmacotherapy = Biomedecine & Pharmacotherapie*.

[22] Santos-Ledo A., Jenny A., Marlow F. L. (2013). Comparative gene expression analysis of the fmnl family of formins during zebrafish development and implications for tissue specific functions. *Gene Expression Patterns*.

[23] Ma G., Wang Z., Liu J. (2021). Quantitative proteomic analysis reveals sophisticated metabolic alteration and identifies FMNL1 as a prognostic marker in clear cell renal cell carcinoma. *Journal of Cancer*.

[24] Chen W. H., Cai M. Y., Zhang J. X. (2018). FMNL1 mediates nasopharyngeal carcinoma cell aggressiveness by epigenetically upregulating MTA1. *Oncogene*.

[25] Zhang M. F., Li Q. L., Yang Y. F., Cao Y., Zhang C. Z. (2020). FMNL1 exhibits pro-metastatic activity via CXCR2 in clear cell renal cell carcinoma. *Frontiers in Oncology*.

[26] Favaro P. M., Traina F., Vassallo J. (2006). High expression of FMNL1 protein in T non-Hodgkin's lymphomas. *Leukemia Research*.

[27] Han Y., Eppinger E., Schuster I. G. (2009). Formin-like 1 (FMNL1) is regulated by N-terminal myristoylation and induces polarized membrane blebbing. *The Journal of Biological Chemistry*.

[28] Katoh A. A., Katoh M. (2003). Identification and characterization of human FMNL1, FMNL2 and FMNL3 genes in silico. *International journal of oncology*.

[29] Miller M. R., Blystone S. D. (2015). Human macrophages utilize the podosome formin FMNL1 for adhesion and migration. *CellBio*.

[30] Miller E. W., Blystone S. D. (2019). The carboxy-terminus of the formin FMNL1ɣ bundles actin to potentiate adenocarcinoma migration. *Journal of Cellular Biochemistry*.

